RETRACTED

# Tooth Loss and the Incidence of Ischemic Stroke and Transient Ischemic Attack: A Systematic Review and Meta-Analysis

**DOI:** 10.1155/2022/1088371

**Published:** 2022-02-14

**Authors:** Tong Guo, Yufen Wang, Qiuming Jiang

**Affiliations:** ^1^School of Basic Medical Sciences, Capital Medical University, Beijing 100069 Beijing, China; ^2^Department of Neurology, The Second Affiliated Hospital of Henan University of Traditional Chinese Medicine, Zhengzhou 450002, Henan, China; ^3^School of Basic Medical Sciences, Capital Medical University, Beijing 100069 Beijing, China

## Abstract

Generally, as the population is aging, ischemic stroke is imposing rising social and economic burdens. On that basis, the early intervention and prevention of ischemic stroke turns out to be a major public health issue. Extensive studies have reached mixed conclusions regarding the correlation between tooth loss and ischemic stroke, as well as transient ischemic attack (TIA). In this paper, a systematic review and meta-analysis is presented where we have aimed to examine whether tooth loss is correlated with a higher incidence of ischemic stroke and TIA in adults. The systematical search was conducted in PubMed, Web of Science, Embase, and The Cochrane library from the inception dates to September 23, 2021, by employing the keywords (i.e., tooth loss and ischemic stroke). Observational studies conducted in adults were included, in which people with and without tooth loss (Exposition and Comparison) were observed to determine the incidence of ischemic stroke/TIA (Outcome). The data were extracted, and the study quality was assessed by two reviewers independently. Moreover, a meta-analysis was conducted to obtain the risk ratios (RRs) and 95% CIs by adopting random-effects models. The major outcome was the incidence of ischemic stroke/TIA in adults with and without tooth loss. On the whole, four cohort studies and three case-control studies were covered, which involved 4,625,514 participants with 33,088 ischemic stroke/TIA cases. In cohort (adjusted RR = 2.58, 95% CI: 2.39–2.79, *P* < 0.00001, *I*^2^ = 31%) and case-control studies (adjusted MD = −4.15, 95% CI: −6.09−(−2.22), *P* < 0.001, *I*^2^ = 77%), a significant correlation was identified between tooth loss and ischemic stroke. The subgroup analyses reported that the results in case-control studies were generally consistent regardless of the selection of controls. This meta-analysis indicated a certain correlation between tooth loss and ischemic stroke.

## 1. Introduction

Stroke refers to the second most common cause of death worldwide, ranking only behind ischemic heart disease [1]. Among all described cases, ischemic stroke takes up to 80–85% [2, 3], which triggers 4.4–4.7 million deaths globally. The etiology of ischemic stroke comprises genetic and environmental factors, thereby elucidating the possibility of early intervention of cerebral ischemia.

RETRACTED

Oral health is associated with the normal function of a wide range of organs and the homeostasis of the whole human body. Periodontal diseases (e.g., periodontitis and dental caries) and tooth loss are considered two common conditions of the oral cavity, thereby significantly impacting the quality of life [4].

Emerging evidence has reported the correlation between poor oral health and an elevated risk of cerebrovascular diseases [5–8], probably attributed to the chronic and systematic inflammation originating from the periodontal infection [9, 10]. However, under unclear causality, results of cohort and case-control studies that assessed the correlation between tooth loss and ischemic stroke were suggested to be conflicting [11, 12]. For this reason, this meta-analysis was conducted to examine the correlation between tooth loss and ischemic stroke.

Generally, as the population is aging, ischemic stroke is imposing rising social and economic burdens. On that basis, the early intervention and prevention of ischemic stroke turn out to be a major public health issue. Extensive studies have reached mixed conclusions regarding the correlation between tooth loss and ischemic stroke. In this paper, a systematic review and meta-analysis are presented where we have aimed to examine whether tooth loss is correlated with a higher incidence of ischemic stroke in adults. The systematic search was conducted in PubMed, Web of Science, Embase, and The Cochrane library from the inception dates to September 23, 2021, by employing the keywords (i.e., tooth loss and ischemic stroke). Observational studies conducted in adults were included, in which people with and without tooth loss (Exposition and Comparison) were observed to determine the incidence of ischemic stroke/transient ischemic attack (Outcome). The data were extracted, and the study quality was assessed by two reviewers independently. Moreover, a meta-analysis was conducted to obtain the risk ratios (RRs) and 95% CIs by adopting random-effects models. The major outcome was the incidence of ischemic stroke/transient ischemic attack in adults with and without tooth loss.

The rest of the manuscript is organized as given below.

In the subsequent section, i.e., Section 2, the proposed meta-analysis and systematic review process is described in detail, along with a detailed discussion of how the mechanism is carried out and which subjects are selected for the successful completion of the proposed study. Various results are presented in Section 3 of the manuscript, which is followed by a brief description of how the problem is identified and how the proposed scheme is effective in resolving the issue. Finally, concluding remarks along with possible future directives are provided.

RETRACTED

## 2. Proposed Analysis Method

### 2.1. Protocol

The present systematic review and meta-analysis were registered at the International Prospective Register of Systematic Reviews (PROSPERO) under the code CRD42021281633 and conducted in accordance with the Preferred Reporting Items for Systematic Reviews and Meta-Analyses (PRISMA) [13].

### 2.2. Search Strategy

Two researchers (i.e., GT and WYF) searched PubMed, EMbase, Web of Science, and the Cochrane library from their inceptions to September 23, 2021, in English by exploiting the main search terms (i.e., “tooth loss” and “ischemic stroke”). The medical subject heading (MeSH) terms and the entry terms were applied in PubMed, and Emtree terms were employed in EMbase. Furthermore, the references of relevant studies for additional studies suit for this meta-analysis were manually checked. The specific search strategy is presented in Supplementary materials.

### 2.3. Selection Criteria

Studies satisfying the following criteria were included:

1. Studies investigating a correlation between tooth loss and the incidence of ischemic stroke
2. Studies including a cohort, case-control, or cross-sectional design and were published in a peer-reviewed journal
3. Studies reporting unadjusted or adjusted effect estimates (e.g., the hazard ratio (HR), the risk ratio (RR), the odds ratio (OR), the incidence rate ratio (IRR), or the standardized incidence ratio (SIR) with corresponding 95% confidence interval (CI), or results allowing for calculating RRs or ORs)

Studies including the conditions below were excluded:

1. Case reports, conference abstracts, letters, reviews, and editorials
2. A retrospective design without a control group
3. Studies assessed based on the Newcastle–Ottawa Scale (NOS) to have scores of less than 7

With two investigators (i.e., GT and WYF) searching and selecting studies independently, any divergence in the meta-analysis was addressed through discussion of all investigators.

### 2.4. Data Extraction

Two investigators (i.e., GT and WYF) independently extracted the information below: author, publication year, study design, country, study period, and the characteristics exhibited by study population (e.g., sample size, sex, and age). Furthermore, the studies ascertaining exposures and outcomes, risk estimates, and adjustment variables were extracted [14]. This process was checked by third evaluators for any disagreement (JQM). If vital data were not available, study authors would also be contacted.

RETRACTED

### 2.5. Quality Assessment of Included Studies

Newcastle-Ottawa Quality Assessment Scale (NOS) was adopted to assess the risk of bias [15]. This scale assessed the risk of bias in several aspects, i.e., the selection of study groups, the comparability of the groups, and the ascertainment of exposures, as well as outcomes. With a maximal total score of 9, the studies were rated to have a high, moderate, or low risk of bias with scores of less than 7, 7 or 8, or 9, respectively. The mentioned process was conducted independently by GT and WYF and then checked by a third examiner (JQM) under any disagreements.

### 2.6. Statistical Analysis

The overall risk of correlation between tooth loss and ischemic stroke was recognized as the primary outcome of interest, whereas others were considered to be secondary. To analyze the data quantitatively and present the results with forest plots, RevMan software (Review Manager v. 5.4.1, The Cochrane Collaboration; Copenhagen, Denmark) was adopted to assess the outcome measures. By complying with the risk estimates of the studies included, the DerSimonian and Laird random-effects model [16] were exploited to determine the pooled RR with 95% CI. RR, HR, and OR were considered to be equivalent [17]. To identify the heterogeneity, Cochran's *Q* test (significance level at *P* < 0.1) was performed in combination with *I*^2^ values for quantification. *I*^2^ < 25%, 25–50%, 51–75%, and >75% were, respectively, considered as no, mild, moderate, and large heterogeneity [18]. Furthermore, subgroup analyses were conducted to verify the proposed hypotheses of heterogeneity. For sensitivity analyses, leave-one-out analyses were also conducted to assess the stability of results.

### 2.7. Certainty of Evidence

The Grading of Recommendations Assessment, Development, and Evaluation (GRADE) approach was adopted to assess the overall certainty of evidence. We evaluated each GRADE item (i.e., study limitations, inconsistency, indirectness, imprecision, and publication bias) for meta-analysis methodology. The level of evidence of observational studies is defined as “low” initially. If there are serious issues related to the above items, the level of evidence will decrease to “very low.” However, it will increase if a strong association or a dose-response gradient is present.

## 3. Results and Evaluations

### 3.1. Study Selection

Our literature search yielded 151 records from the mentioned databases. After removing duplicates, 109 studies had their titles and abstracts assessed, of which 39 studies were assessed by reading their full texts. Ultimately, seven studies complied with the inclusion criteria for this review (Figure 1).

RETRACTED

### 3.2. Study Characteristics

Of the seven selected studies, four carried out the prospective cohort studies [6, 11, 19, 20], and three pertained to case-control studies [21–23]. The studies were conducted in the United States (*n* = 2), Germany (*n* = 2), Korea (*n* = 1), Australia (*n* = 1), and Brazil (*n* = 1). The sample size ranged from 183 to 4,404,970.  Table 1 lists other population characteristics.

Dental examination and self-reported questionnaires were generally adopted to assess edentulism or tooth loss in the seven included studies [6, 11, 19–23], while one study [23] also selected a structured questionnaire to interview the participants for their tooth numbers. Likewise, six of the seven included studies assessed ischemic stroke via medical evaluation, while Wu et al. [20] chose to review the medical history. Three studies [6, 11, 19] only included ischemic stroke, one [20] assessed both ischemic and hemorrhagic stroke, and the other three studies [21–23] were concerned with ischemic stroke and transient ischemic attack (TIA). Although TIA may not result in permanent neurological deficits, those affected would be at a higher risk for subsequent ischemic events [24], so the incidence of ischemic stroke and TIA were combined in the quantitative analysis (Table 2).

### 3.3. Quality Assessment of Included Studies

Tables 3 and 4 list NOS scores of the included studies. Quality scores of the eight studies for qualitative analysis ranged from 6 to 9. One study was rated as low risk of bias, six studies as moderate, and one study as high. The cohort study by Choe et al. [25] only included employed people and their families from a national insurance plan, which might underrepresent those unemployed. When ascertaining the fatal outcomes of ischemic stroke, it searched the death certificates, increasing the false-positive rate due to the possible misclassification. Besides, a self-reported questionnaire without validation might not adjust the results completely for other risk factors. Thus, we finally excluded this Korean cohort study for meta-analysis due to its high risk of bias.

### 3.4. Analysis of Outcomes

In cohort studies, Risk Ratio (RR), the Hazard ratio (HR), and Odds Ratio (OR) were adopted to indicate the level of correlation between tooth loss and ischemic stroke. Most of these ratios also reported the risk estimates with different numbers of teeth, while Wu et al. [20] only presented the RR in edentulous participants. According to case-control studies, only Grau et al. [21] provided the ORs for the respective range of teeth numbers, while others only presented the teeth numbers in cases and controls, together with the P-values (Table 2).

RETRACTED

Tooth loss is significantly correlated with a higher risk of ischemic stroke in the cohort (adjusted RR = 2.58, 95% CI: 2.39–2.79, *I*^2^ = 31%; Figure 2) and case-control studies (adjusted MD = −4.15, 95% CI: −6.09−(−2.22), *P* < 0.001, *I*^2^ = 77%; Figure 3). Heterogeneity across the cohort studies was mild, while significant heterogeneity was observed across the case-control studies. However, removing the study, Leao et al. [22] revealed significantly lower heterogeneity for case-control studies (adjusted MD = −3.38, 95% CI: −4.41−(−2.35), *I*^2^ = 23.6%; Figure 4).

Since the selection of controls was not consistent in three case-control studies, a subgroup analysis was conducted (Figure 5). The pooled adjusted MD for cases VS hospital controls reached −4.67 (95% CI: −8.76−(−0.57), *P*=0.03, *I*^2^ = 91%), and the pooled adjusted MD for cases VS population controls was −3.83 (95% CI: −5.11−(−2.54), *P* < 0.00001, *I*^2^ = 0%). No heterogeneity was observed in the second subgroup, while the heterogeneity across studies included in the first subgroup was noticeably greater. As revealed from this meta-analysis, no difference in the selection of controls was observed.

Since the approaches to adjust confounding factors varied with studies, a sensitivity analysis was conducted to confirm robustness by excluding individual study estimates once to determine the effect of the respective study. The omission of any one study did not significantly alter the pooled RR, and the estimate in the respective case was well within the confidence limits of the overall RR.

### 3.5. Publication Bias

No clear publishing bias was identified by complying with the funnel plots (Figures 6 and 7) for cohort and case-control studies.

### 3.6. Assessment of the Level of Evidence (GRADE)

A total of seven studies were evaluated for the level of evidence for the association between tooth loss and ischemic stroke (Table 5). Evidence in four cohort studies [6, 11, 19, 20] was rated as high due to the large effect (RR > 2) and dose-response gradient. However, evidence in three case-control studies [21–23] was classified as low due to the problems in inconsistency.

## 4. Discussion

According to the results of this meta-analysis, a correlation was revealed between tooth loss and the incidence of ischemic stroke, which complied with four cohort studies and three case-control studies. To be specific, there were 4,625,514 participants in total, which involved 33,088 ischemic stroke/TIA cases. In addition, consistent findings were also indicated in the subgroup analysis by selecting controls.

RETRACTED

Several mechanisms are likely to clarify the correlation between tooth loss and ischemic stroke.

- Tooth loss is generally considered as the ultimate stage of periodontal diseases (e.g., periodontitis), which is indicated to be associated with ischemic stroke via chronic inflammation [26]. Upregulated levels of proinflammatory cytokines attributed to the inflammation in the oral cavity can be transmitted to the central nervous system via blood circulation, thereby inducing endothelial dysfunction [27]. For instance, C - reactive protein and IL-6 act as indicators of increased stroke risk and the biomarkers of periodontitis and subsequent tooth loss [28–31].
- Tooth loss is able to be attributed to dental caries, and excessive intake of carbohydrates primarily causes dental caries. As revealed from existing evidence, increased carbohydrate intake is associated with an elevated risk of stroke, so an indirect relationship exists between tooth loss and stroke [32]. Third, tooth loss is constantly accompanied by and induces the disruption of periodontal tissue integrity, thereby facilitating the translocation of oral microbiota and the consequent systematic inflammation. Inflammatory lesion of vascular endothelial cells shows a correlation with an upregulated risk of ischemic stroke [33, 34].

Several factors were found to limit the interpretation of this review. First, there were significant differences in the criteria adopted to stratify the samples into groups according to their teeth number, which might markedly increase the heterogeneity of the pooled studies, thereby making the results questionable. Across the case-control studies, *I*^2^ index exceeded 70%, probably attributed to the study design, which involved the definition and selection of participants and the inherent retrospective design. By removing the study by Leao et al. [22], the heterogeneity decreased markedly, with *I*^2^ index altered into 23.6%. Second, the unmeasured bias attributed to the combination of various individual studies might reduce the quality of this meta-analysis. The study by Choe et al. [25] was considered with a high risk of bias, in which the data were collected from an insurance plan covering employed people and their families, thereby underrepresenting Koreans without jobs. Besides, the fatal ischemic stroke was ascertained by searching the death certificates, which might upregulate the false-positive rates. Thus, the mentioned study was removed to address this problem. Third, as impacted by the limited numbers of ischemic stroke cases in the included studies, more large-scale and well-designed epidemiological studies focusing on the correlation between tooth loss and ischemic stroke are warranted.

RETRACTED

## 5. Conclusion

Generally, as the population is aging, ischemic stroke is imposing rising social and economic burdens. On that basis, the early intervention and prevention of ischemic stroke turn out to be a major public health issue. Extensive studies have reached mixed conclusions regarding the correlation between tooth loss and ischemic stroke. In this paper, a systematic review and meta-analysis are presented where we have aimed to examine whether tooth loss is correlated with a higher incidence of ischemic stroke in adults. The systematic search was conducted in PubMed, Web of Science, Embase, and The Cochrane library from the inception dates to September 23, 2021, by employing the keywords (i.e., tooth loss and ischemic stroke). Observational studies conducted in adults were included, in which people with and without tooth loss (Exposition and Comparison) were observed to determine the incidence of ischemic stroke/transient ischemic attack (Outcome). The data were extracted, and the study quality was assessed by two reviewers independently. Moreover, a meta-analysis was conducted to obtain the risk ratios (RRs) and 95% CIs by adopting random-effects models. The major outcome was the incidence of ischemic stroke/transient ischemic attack in adults with and without tooth loss. The results of this meta-analysis suggest a certain correlation between tooth loss and ischemic stroke in adults, which highlights the need to place more focus on the risk of ischemic stroke in edentulous people and the possibility of early intervention or even prevention of cerebral ischemia. However, given the low certainty of the mentioned results and limited amounts of ischemic stroke cases, more high-quality studies should be involved.

## Figures and Tables

**Figure 1:** Flowchart of literature searching and selection, according to the PRISMA statement.

**Figure 2:** Forest plot for meta-analysis of tooth loss and ischemic stroke in cohort studies.

**Figure 3:** Forest plot for meta-analysis of tooth loss and ischemic stroke in case-control studies.

**Figure 4:** Forest plot for meta-analysis of tooth loss and ischemic stroke in case-control studies (after removing the study with high heterogeneity).

**Figure 5:** Forest plot for subgroup analysis of tooth loss and ischemic stroke in case-control studies, according to the selection of controls.

**Figure 6:** Funnel plots of tooth loss and ischemic stroke in cohort studies.

**Figure 7:** Funnel plots of tooth loss and ischemic stroke in case-control studies.

**Table 1:** Characteristics of studies included in the meta-analysis of tooth loss in relation to incidence of ischemic stroke.

Author (year)	Study design	Country	Study period	Study population	Sex	Age at baseline (years)	NOS scores
Wu et al. (2000)	Cohort	USA	1971–1992	Total: 9,962	Mix	25–74	8
				Dentate: 7,780 (including no periodontal disease: 3634)			
				Edentulous: 2,182			
Joshipura et al. (2003)	Cohort	USA	1986–1998	Total: 41,380	Male	40–75	8
				25–32 teeth: 34,767			
				17–24 teeth: 4,527			
				11–16 teeth: 903			
				0–10 teeth: 1183			
Joshy et al. (2016)	Cohort	Australia	2006–2011	Total: 167,697	Mix	45–75	7
				≥20 teeth: 117,464			
				10–19 teeth: 30,013			
				1–9 teeth; 11,423			
				None: 8,797			
Lee et al. (2019)	Cohort	Korea	2007–2016	Total: 4,404,970	Mix	≥20	9
				28 teeth: 3,978,654			
				24–27 teeth: 329,461			
				14–23 teeth: 81,337			
				1–13 teeth: 12,601			
				None: 2,917			
Grau et al. (2004)	Case-control	Germany	1998–2000	Total: 771	Mix	18–75	7
				Cases: 303			
				Population controls: 168			
				Hospital controls: 300			
Palm et al. (2014)	Case-control	Germany	2010–2011	Total: 183	Mix	18–80	8
				Cases: 96			
				Population controls: 87			
Leao et al. (2021)	Case-control	Brazil	2015–2018	Total: 458	Mix	＞0	7
				Cases: 229			
				Hospital controls: 229			

RETRACTED

**Table 2:** Exposures, outcomes, and adjustment variables of seven included studies of tooth loss in relation to incidence of ischemic stroke.

Author (year)	Tooth loss evaluation	Ischemic stroke assessment	Effect estimates	Risk	Adjustment variables
Wu et al. (2000)	Dental examination	Review of medical history, including ischemic and hemorrhagic stroke	RR	No periodontal disease: 1.00^R^	Age, sex, race, education, poverty index, diabetes status, hypertension, smoking status, average alcohol use, body mass index, and serum cholesterol
				Edentulous: 1.41 (0.96–2.06)	
Joshipura et al. (2003)	Self-reported questionnaire	Medical evaluation and self-reports, only including ischemic stroke	HR	25–32 teeth: 1.00^R^	Age, smoking, alcohol consumptions, body mass index, physical activity, family history of myocardial infarction, multivitamin supplement use, vitamin E use, history of hypertension, diabetes, hypercholesterolemia, and professions
				17–24 teeth: 1.50 (1.14–1.97)	
				11–16 teeth: 1.74 (1.08–2.81)	
				0–10 teeth:1.66 (1.10–2.51)	
Joshy et al. (2016)	Self-reported questionnaire	Medical evaluation and self-reports, only including ischemic stroke	HR	20 teeth: 1^R^	Age, sex, tobacco smoking, alcohol consumption, Australian born status, region of residence, education, health insurance, physical activity, and body mass index
				10–19 teeth: 1.11 (0.72–1.73)	
				1–9 teeth: 0.90 (0.59–1.40)	
				None: 1.20 (0.90–1.62)	
Lee et al. (2019)	Dental examination	Medical evaluation, only including ischemic stroke	HR	28 teeth: 1^R^	Age, sex, body mass index, diagnosis of diabetes mellitus, hypertension, dyslipidemia, chronic pulmonary disease, end-stage renal disease, smoking history, drinking history, exercise habits, and low income level
				24–27 teeth: 1.12 (1.09–1.16)	
				14–23 teeth: 1.26 (1.20–1.32)	
				1–13 teeth: 1.28 (1.18–1.39)	
				None: 1.30 (1.13–1.50)	
				Total: 1.015 (1.012–1.018)	
Grau et al. (2004)	Dental examination	Medical evaluation, including ischemic stroke and transient ischemic attack	OR	No tooth loss: 1.0^R^	Age and sex
				1–19 teeth loss: 0.97 (0.42–2.2)	
				20–27 teeth loss: 0.75 (0.27–2.05)	
				All teeth loss: 1.50 (0.52–4.44)	
Palm et al. (2014)	Dental examination and interview using a structured questionnaire	Medical evaluation, self-reports and review of medical history, including ischemic stroke and transient ischemic attack	*P*-value	Teeth number	None
				Cases: 13.8 ± 10.8	
				Population controls: 16.6 ± 10.1	
				*P*-value: 0.04	
Leao et al. (2021)	Dental examination	Medical evaluation, including ischemic stroke and transient ischemic attack	*P*-value	Teeth number	None
				Cases: 11.78 ± 10.06	
				Hospital controls: 18.53 ± 8.02	
				*P*-value: <0.01	

RETRACTED

**Table 3:** Newcastle-Ottawa quality assessment scale for cohort studies.

Cohort study	Selection				Comparability	Outcome			Total
	1	2	3	4		1	2	3	
Joshipura et al. (2003)	★	★	☆	★	★★	★	★	★	8
Joshy et al. (2016)	★	★	☆	★	★★	★	☆	★	7
Lee et al. (2019)	★	★	★	★	★★	★	★	★	9
Wu et al. (2000)	★	☆	★	★	★★	★	★	★	8

**Table 4:** Newcastle-ottawa quality assessment scale for case-control studies.

Case-control study	Selection				Comparability	Exposure			Total
	1	2	3	4		1	2	3	
Grau et al. (2004)	★	★	☆	★	★★	★	★	☆	7
Leao et al. (2021)	★	★	☆	★	★★	★	☆	★	7
Palm et al. (2014)	☆	★	★	★	★★	★	★	★	8

**Table 5:** Grade evidence profile: Association between tooth loss and ischemic stroke.

Certainty assessment							Summary of findings				Certainty
							№ of patients		Effect		
No of studies	Study design	Risk of bias	Inconsistency	Indirectness	Imprecision	Other considerations	Tooth loss	Control	Relative soft-enter (95% CI)	Absolute soft-enter (95% CI)	
4	Cohort studies	Not serious	Not serious	Not serious	Not serious	Strong association, soft-enter dose response gradient	7290/485134 (1.5%)	24867/4138665 (0.6%)	**RR 2.58** soft-enter (2.39 to 2.79)	**9 more per 1,000** soft-enter (from 8 more to 11 more)	⊕⊕⊕⊕
											High
3	Case-control studies	Not serious	Serious^a^	Not serious	Not serious	Strong association	931 cases 784 controls		**MD-4.15** soft-enter (−6.09 to −2.22)	**0 fewer per 1,000** soft-enter (from 0 fewer to 0 fewer)	⊕⊕○○
											Low
							—	0%			

Notes: a. Considerable heterogeneity (I^2^ = 77%). **A**bbreviations: CI: confidence interval; RR: risk ratio.

RETRACTED

## Data Availability

The data underlying the results presented in the study are included within the manuscript.

## Supplementary Materials

Supplementary Materials Search strategy.
